The article "LncRNA SBF2-AS1 Facilitates Nonsmall Cell Lung Cancer Progression by Targeting miR-520a-3p" was retracted in 2023. Reasons: signs of a paper mill; suspected computer-generated content; unreliable results or conclusions; concerns about the data.

# LncRNA SBF2-AS1 Facilitates Nonsmall Cell Lung Cancer Progression by Targeting miR-520a-3p

**DOI:** 10.1155/2022/2223149

**Published:** 2022-04-11

**Authors:** Yi Wang, Yanzhi Zou, Qingmei Zhang, Defu Chen, Lin Lin

**Affiliations:** ^1^Department of Respiration, The People's Hospital of Zhangqiu Area, Jinan 250200, China; ^2^Occupational Disease Department, The Second Affiliated Hospital of Shandong University of Traditional Chinese Medicine, Jinan 250001, China; ^3^Emergency Ward, Qingdao Hospital of Traditional Chinese Medicine, Hiser Medical Group of Qingdao, Qingdao 266033, China; ^4^Department of Cardio-Thoracic Surgery, Zhangqiu District People's Hospital, Jinan 250200, China; ^5^No. 1 Department of Respiratory and Critical Care Medicine, Shengjing Hospital of China Medical University, Shenyang 110004, China

## Abstract

**Background:**

Long noncoding RNA (lncRNA) SET-binding factor 2 (SBF2) antisense RNA1 (SBF2-AS1), which acts as an oncogene in various cancers, can promote tumors progression. The study aimed to explore the role and molecular mechanism of SBF2-AS1 in nonsmall cell lung cancer (NSCLC).

**Methods:**

qRT-PCR was introduced to detect SBF2-AS1 and miR-520a-3p expression in NSCLC. The effects of SBF2-AS1 and miR-520a-3p on the proliferation, migration, and invasion of NSCLC cells were assessed through cell counting kit-8 (CCK-8) and transwell assay. Furthermore, the relationship of SBF2-AS1 and miR-520a-3p was verified by the RNA immunoprecipitation (RIP) assay, dual-luciferase assay, and Spearman correlation analysis.

**Results:**

In NSCLC tissues, SBF2-AS1 was highly expressed, while miR-520a-3p expression has decreased. The overall survival of NSCLC patients with high SBF2-AS1 expression was lower. SBF2-AS1 silencing repressed the proliferation, migration, and invasion of NSCLC cells. SBF2-AS1 directly interacted with miR-520a-3p, and a negative relationship was observed between their expression levels in NSCLC tissues. More importantly, the suppression of SBF2-AS1 silencing on the proliferation, migration, and invasion in NSCLC cells was counteracted by miR-520a-3p inhibition.

**Conclusion:**

SBF2-AS1 accelerated the proliferation, migration, and invasion of NSCLC cells via mediating miR-520a-3p, thus promoting NSCLC progression.

## 1. Introduction

Lung cancer (LC) is one of the cancers with the highest incidence rate in China and will become the main cause for cancer death [1]. According to the type of pathology, it can be divided into two main types: small cell lung cancer (SCLC) and NSCLC [2, 3]. The 5-year survival rate of NSCLC is low, and the pathogenesis of NSCLC is complex [2, 3]. Many patients are already at the advanced stage when diagnosed and missed the opportunity of surgery because of metastasis occurring. Currently, the comprehensive application of surgical, chemotherapy, radiotherapy, and other treatment methods has obtained remarkable achievements, but their long-term benefits are limited [4, 5]. Therefore, the immediate priority is to further explore molecular mechanisms of NSCLC progression. Many lncRNAs are found to be associated with various processes of gene regulation, which is related to the occurrence and development of NSCLC [6]. At present, the research of lncRNA in NSCLC has only uncovered a small part of the mystery, and more biological functions and specific molecular mechanisms are still unknown.

SBF2-AS1 is located on chromosome 11p15.4 and is a member of a novel lncRNA family [7]. SBF2-AS1 is upregulated in esophageal squamous cell carcinoma (ESCC), cervical cancer (CC), hepatocellular carcinoma (HCC), and osteosarcoma (OS) to promote the development of cancer, and its expression is associated with poor prognosis [7–10]. SBF2-AS1 expression is distinctly increased, and its silencing represses proliferation and invasion of ESCC [8]. In CC, abnormal expression of SBF2-AS1 promotes its progression through the regulation of miR-361-5p/FOXM1 axis [9]. Moreover, SBF2-AS1 regulates TGF-BR1 through sponging miR-140-5p to participate in the progression of HCC [7]. Besides, the expression of miR-30a and FOXA1 is regulated by SBF2-AS1 silencing to suppress the malignant biological behavior of OC cells [10]. Similarly, SBF2-AS1 acts as an oncogene in LC, and its upregulation can promote cell proliferation and metastasis, reduce the sensitivity of radiotherapy, inhibit apoptosis, and is closely related to unfavorable prognosis [11–13]. The discovery and elucidation of SBF2-AS1 function provides a new molecular marker for the diagnosis and prognosis of NSCLC, as well as a potential therapeutic target. Nevertheless, the specific regulation mechanism still needs to be further clarified.

Thus, we investigated SBF2-AS1's functions in NSCLC. It further proved whether SBF2-AS1 could regulate miR-520a-3p expression to mediate the NSCLC cells malignant biological behavior, thereby revealing the mechanism of NSCLC progression and providing new targets for NSCLC-targeted therapy and research directions.

## 2. Materials and Methods

### 2.1. Clinical Samples

Thirty-six cases of NSCLC patients admitted to People's Hospital of Zhangqiu Area and confirmed by surgery and pathology were selected. Inclusion criteria: patients diagnosed with NSCLC confirmed by surgical pathology, patients did not receive chemotherapy or molecular targeted therapy before surgery, and case information is complete. Exclusion criteria: severe organ dysfunction, patients with other chronic diseases (diabetes and coronary heart disease), and patients with chronic obstructive pulmonary disease, asthma, tuberculosis, and other lung diseases. The tumor was surgically removed, and the adjacent tissues were removed during the operation. Informed consent form was obtained from all patients. This study was endorsed by the Ethics Committee of People's Hospital of Zhangqiu Area.

### 2.2. Cell Culture

The normal human bronchial epithelial cell (16HBE) and four NSCLC cells (A549, Calu-3, HCC827 and PC9) were obtained from Shanghai Cell Bank and ATCC. All cells were cultured in DMEM containing 10% FBS (Invitrogen, USA) at 37°C with 5% CO_2_.

### 2.3. Cell Transfections

Cells in the logarithmic growth phase were cultured with 3 × 10^5^ cells/well. When the cells were about 60–70% fused, si-SBF2-AS1 (small interfering RNA of SBF2-AS1), miR-520a-3p inhibitor (inhibitor), miR-520a-3p mimic (mimic), and their control (anti-NC or miR-NC), obtained from GenePharma in Shanghai, were transfected with Lipofectamine 2000 (Invitrogen, USA). After transfected cells were cultured for 24 h, the levels of RNA were detected to verify the transfection efficiency and continue related experiments.

### 2.4. CCK-8 Assay

The transfected cells were inoculated on a 96-well plate with 2 × 10^3^ cells/well. At 24, 48, 72, and 96 h after cell inoculation, CCK-8 solution (Dojindo, Japan) was added and mixed gently. Culture was continued for 2 h in an incubator at 37°C. The 450 nm absorbance was detected by the microplate reader (Bio-Rad, Carlsbad, CA).

### 2.5. Transwell Assay

The cell density of each group was adjusted into 1 × 10^5^ cells/ml. The upper chamber was inserted with 100 *μ*l cell suspension, and 600 *μ*l serum-containing medium was filled with lower chamber. The cells were routinely cultured overnight. Subsequently, the moved cells were fixed with 4% paraformaldehyde and stained with 0.1% crystal violet. The migrated cells were observed under the microscope.

In the cell invasion experiment, upper chamber was precoated with Matrigel (BD Biosciences, USA). The following procedures were the same as above. Finally, 5 randomly fields were selected to count the number of invaded cells.

### 2.6. Dual-Luciferase Reporter Assay

The binding sites of SBF2-AS1 and miR-520a-3p were predicted by bioinformatics analysis using ENCORI (The Encyclopedia of RNA Interactomes) online (https://starbase.sysu.edu.cn/index.php). All parameters were default. The binding fragment was amplified and inserted into the luciferase vector to construct the wild-type plasmid of SBF2-AS1 (SBF2-AS1-wt); then, the binding site was mutated to construct the mutant-type plasmid of SBF2-AS1 (SBF2-AS1-mut). The transfection was performed as previously mentioned. Luciferase activity was detected by the dual-luciferase reporter kit (Promega, USA).

### 2.7. RIP Assay

The collected cells were lysed by RIP lysate, and the supernatant was centrifuged. According to the instruction of the RIP^TM^ kit (Millipore, USA), immunoprecipitation buffer (containing ribonuclease inhibitor, protease inhibitor, and deoxyribonuclease) and cell lysate were added to EP tubes containing magnetic beads. Then, the mixture was incubated with IgG or Ago2 antibody (Abcam, USA) at 4°C overnight, and the supernatant was discarded by centrifugation. Finally, the RNA was purified and dissolved. The expressions of RNAs were detected by qRT-PCR. The group without antibody was the positive control group (input), the group with IgG antibody was the negative control group (IgG), and the group with Ago2 antibody was the experimental group (Ago2).

### 2.8. qRT-PCR

Total RNA was extracted by the TRIzol kit (Invitrogen, USA). The qualified RNA was selected for subsequent experiments. CDNA was synthesized using the Super Master Mix synthesis kit (TaKaRa, Japan), with 50 *μ*g total RNA as the template. qRT-PCR was performed on the ABI 7300 System (Applied Biosystems, USA) according to the SYBR Real-Time PCR kit (TaKaRa, Japan) instructions. 2^−ΔΔCt^ was used to express the relative expressions of SBF2-AS1 or miR-520a-3p with U6 or GAPDH as the internal reference. Primers are given in Table 1.

### 2.9. Statistical Analysis

Data were expressed as mean ± SD. Statistical analysis between two groups was performed by the GraphPad Prism 5.0 software. *P* < 0.05 was indicated a statistically significant.

## 3. Results

### 3.1. Abnormal Expression of SBF2-AS1 in NSCLC Tissues and Cells

SBF2-AS1 expression in 36 cases NSCLC tissues was detected, and its expression in NSCLC tissues was obviously enhanced (Figure 1(a)). At the same time, SBF2-AS1 expression in four NSCLC lines A549, Calu-3, HCC827, and PC9 was increased versus 16HBE cells (Figure 1(b)). Moreover, SBF2-AS1 expression in A549 and Calu-3 cells was higher than that in HCC827 and PC9 cells (Figure 1(b)). On the basis of above results, A549 and Calu-3 cells were selected to conduct the functional experiments.

Based on the average expression of SBF2-AS1 (2.275) in patients, they were assigned into the high SBF2-AS1 level group and low SBF2-AS1 level group. There were 18 cases in the high expression group with average expression level of SBF2-AS1 as (3.10 ± 0.66). Eighteen cases of the low expression group are with the average of (1.45 ± 0.47). More importantly, there was a significantly shorter overall survival of patients who had high SBF2-AS1 expression compared to low SBF2-AS1 expression (Figure 1(c)).

### 3.2. SBF2-AS1 Knockdown Inhibits Cellular Malignancy

A549 and Calu-3 cells were selected for the transfection with si-SBF2-AS1 to investigate the role of SBF2-AS1 in NSCLC progression. After transfection, the relative expression of SBF2-AS1 was decreased by si-SBF2-AS1 (Figures 2(a) and 2(b)), indicating that transfection had been successful and subsequent experiments could be performed. Cell proliferation was detected by CCK-8 assay. The proliferation of A549 and Calu-3 cells was decreased after transfection with si-SBF2-AS1, indicating that SBF2-AS1 knockdown could inhibit the proliferation of NSCLC cells (Figures 2(c) and 2(d)). Transwell experiment results are shown in Figures 2(e)–2(h). The number of invaded and migrated A549 and Calu-3 cells transfected with si-SBF2-AS1 was also decreased. Collectively, SBF2-AS1 silencing inhibited NSCLC cell proliferation, invasion, and migration and further proved that SBF2-AS1 could promote NSCLC progression.

### 3.3. MiR-520a-3p Directly Binds to SBF2-AS1

Bioinformatics analysis found that miR-520a-3p could bind to the complementary sequence of SBF2-AS1 (Figure 3(a)). Later, dual-luciferase reporter experiments were used to further explore the targeting relationship between SBF2-AS1 and miR-520a-3p. The results showed that luciferase activity was significantly inhibited in the presence of miR-520a-3p mimic and SBF2-AS1-wt, but there was no change of other groups (Figure 3(b)). Similarly results were observed in the RIP experiment. Compared with the IgG group, SBF2-AS1 and miR-520a-3p were enriched in the Ago2 group and input group, and the expression of the input group was higher than that in the Ago2 group (Figure 3(c)). It was confirmed that SBF2-AS1 could interact with miR-520a-3p through complementary binding sites. The regulatory relationship between SBF2-AS1 and miR-520a-3p was further examined. It was found that miR-520a-3p expression was increased by SBF2-AS1 silencing, but decreased in the presence of SBF2-AS1 overexpressing (Figure 3(d)). It proposed that SBF2-AS1 could negative regulate miR-520a-3p.

### 3.4. MiR-520a-3p Was Downexpressed and Negatively Correlated with SBF2-AS1 Expression in NSCLC

After clarifying the regulatory relationship between SBF2-AS1 and miR-520a-3p, we detected miR-520a-3p expression levels in NSCLC tissues and cells, respectively. It was found that miR-520a-3p expression was decreased in NSCLC tissues (Figure 4(a)). The same expression trend was also exhibited in NSCLC cells (Figure 4(b)). More importantly, miR-520a-3p expression showed a significant negative correlation with SBF2-AS1 expression in tissues (Figure 4(c)).

### 3.5. SBF2-AS1 May Regulate NSCLC Cellular Malignancy through miR-520a-3p

To explore whether SBF2-AS1 regulated cell biological behavior by miR-520a-3p, si-SBF2-AS1 and miR-520a-3p inhibitors were cotransfected into NSCLC cell. On the basis of above experiments, the miR-520a-3p inhibitor was transfected into NSCLC cells to decrease its expression (Figure 5(a)). Then, the rescue experiment including CCK-8 and transwell assay was introduced. CCK-8 assay revealed that the inhibition of si-SBF2-AS1 on NSCLC cells proliferation was relieved by the cotransfection of the miR-520a-3p inhibitor (Figure 5(b)). In transwell assays, we found that suppression of miR-520a-3p could reverse the cell migration and invasion capacities hampered by SBF2-AS1 silencing (Figures 5(c) and 5(d)). Collectively, we found that suppression of miR-520a-3p weakened the inhibition of NSCLC cells proliferation, invasion, and migration abilities caused by SBF2-AS1 knockdown, suggesting SBF2-AS1 might play a promoting role in NSCLC by targeting miR-520a-3p.

## 4. Discussion

Numerous lncRNAs are dysregulated in NSCLC and regulated multiple biological processes through various miRNAs and genes [6]. Therefore, the construction of lncRNA-mediated regulatory networks and signal pathway networks will reveal the molecular mechanism of lncRNA in NSCLC progression. Now, SBF2-AS1's role in NSCLC was explored.

SBF2-AS1 was upregulated in multiple cancers. SBF2-AS1 overexpression accelerated cell proliferation ability in NSCLC [11]. Additionally, Zhao et al. found that SBF2-AS1 upregulation has close relationship to NSCLC progression and poor prognosis [12]. Similarly, SBF2-AS1 was also upregulated in NSCLC, and its high expression brought a low overall survival in this study. NSCLC cells proliferation, migration, and invasion abilities were markedly repressed after SBF2-AS1 silencing. Therefore, SBF2-AS1 may play a carcinogenic role in NSCLC.

miR-520a-3p is involved in many normal or abnormal pathophysiological processes, such as cell proliferation, migration, and invasion. miR-520a-3p, as tumor suppressor of many malignant tumors, participates in the occurrence and development of different tumors through targeting the corresponding genes. In breast cancer (BC), miR-520a-3p upregulation inhibits proliferation and metastasis of BC cells by the regulation of CCND1 and CD44 [14]. Besides, miR-520a-3p overexpression suppresses malignant biological behavior of gastric cancer cells by targeting SKA2 [15]. Similar results have been confirmed in papillary thyroid carcinoma (PTC); miR-520a-3p achieves the purpose of suppressing tumor progression through resisting EMT and reducing cell migration and invasion capabilities by regulating the JAK/STAT pathway [16]. However, interactions between lncRNAs and miR-520a-3p are rarely reported in cancers.

In NSCLC, miR-520a-3p as a tumor suppressor was downregulated, and its upregulation impeded tumor progression by regulating MAP3K2, HOXD8, and PI3K/AKT/mTOR pathways [17–19]. What is more, HOXA-AS2, one lncRNA, could target miR-520a-3p, thus regulating HOXD8 and MAP3K2 expressions to accelerate NSCLC progression [20]. Bioinformatics analysis predicted that SBF2-AS1 and miR-520a-3p had binding sequence sites, and there was a regulatory relationship between them. Functional rescue experiments indicated that SBF2-AS1 could target miR-520a-3p and promote the proliferation, migration, and invasion behavior of NSCLC cells, while inhibiting miR-520a-3p expression attenuated the suppression of SBF2-AS1 silencing on NSCLC cells.

In summary, SBF2-AS1 regulated miR-520a-3p expression to affect the cell proliferation, invasion, and migration ability of NSCLC. This research confirmed a new regulatory network of NSCLC cell proliferation, migration, and invasion and will provide corresponding theoretical for understanding the molecular mechanism of NSCLC and exploring new potential treatment strategies. However, the collected clinical cases were not rich enough to fully demonstrate the close relationship between SBF2-AS1 and clinicopathological features. Moreover, we have not explored the regulatory mechanism of the downstream target genes or signaling pathway in SBF2-AS1. Therefore, more clinical cases and experiment results (such as animal experiments, target genes, and pathological data) are needed to improve the research and clarify the network composition of SBF2-AS1.

## 5. Conclusion

In this study, the differential expression of SBF2-AS1 in NSCLC tissues and cells was identified. Subsequently, it was proved that SBF2-AS1 knockdown had a certain inhibitory effect on NSCLC cell proliferation, invasion, and migration ability. The existence of the SBF2-AS1/miR-520a-3p regulatory pathway was identified in NSCLC. Therefore, it may have the potential to be a molecular targeted therapy and a marker to judge the prognosis of NSCLC patients, which provides a new idea for NSCLC treatment in the future.

## Figures and Tables

**Figure 1:** SBF2-AS1's expression in NSCLC was measured by qRT-PCR. (a) SBF2-AS1 expression increased in NSCLC tissues. (b) SBF2-AS1 expression elevated in NSCLC cells. (c) The correlation between SBF2-AS1 expression and overall survival of NSCLC patients analyzed by Kaplan–Meier analysis. ^*∗∗*^*P* < 0.01, ^*∗∗∗*^*P* < 0.001.

**Figure 2:** SBF2-AS1 knockdown repressed cell proliferation, invasion, and migration. ((a), (b)) SBF2-AS1 expression measured in A549 and Calu-3 cells with si-SBF2-AS1 transfection. ((c), (d)) Cells proliferation detected in NSCLC cells with si-SBF2-AS1 transfection by CCK-8 assay. ((e), (f)) Transwell migration assays showed that SBF2-AS1 knockdown reduced the migration of NSCLC cells. ((g), (h)) Transwell invasion assays revealed that inhibition of SBF2-AS1 reduced the invasion of NSCLC cells. ^*∗*^*P* < 0.05, ^*∗∗*^*P* < 0.01.

**Figure 3:** miR-520a-3p directly binds to SBF2-AS1. (a) Binding sites of miR-520a-3p and SBF2-AS1 are presented. (b) Luciferase activity detected in NSCLC cells. (c) SBF2-AS1 and miR-520a-3p enriched by RIP assay determination. (d) The expression of miR-520a-3p in NSCLC cells after transfecting si-SBF2-AS1. ^*∗*^*P* < 0.05, ^*∗∗*^*P* < 0.01.

**Figure 4:** miR-520a-3p expression was reduced and negatively correlated with SBF2-AS1 expression in NSCLC. (a) miR-520a-3p was low expressed in NSCLC tissues. (b) miR-520a-3p expression reduced in NSCLC cells. (c) The relevance of SBF2-AS1 and miR-520a-3p expression. ^*∗∗*^*P* < 0.01.

**Figure 5:** miR-520a-3p reversed the SBF2-AS1 suppressive effect on cellular malignancy in NSCLC. (a) miR-520a-3p expression decreased in NSCLC cells with miR-520a-3p inhibitor transfection. (b) Cell proliferation measured in NSCLC cells after inhibiting both SBF2-AS1 and miR-520a-3p. (c) The effect of SBF2-AS1 knockdown on migration of NSCLC cells could be reversed by the miR-520a-3p inhibitor. (d) The suppressing effects of si-SBF2-AS1 on the invasion of NSCLC cells rescued by the miR-520a-3p inhibitor. ^*∗*^*P* < 0.05, ^*∗∗*^*P* < 0.01.

**Table 1:** Primer sequences for real-time fluorescence quantification PCR.

Gene Name	Primer sequences (5′-3′)
GAPDH	F GCACCGTCAAGGCTGAGAAC
	R TGGTGAAGACGCCAGTGGA

U6	F CTCGCTTCGGCAGCACA
	R AACGCTTCACGAATTTGCGT

SBF2-AS1	F CACGACCCAGAAGGAGTCTAC
	R CCCGGTACCTTCCTGTCATA

miR-520a-3p	F ACACTCCAGCTGGGAAAGTGCTTCCC
	R CTCAACTGGTGTCGT GGA

## Data Availability

The data used to support the findings of this study are available from the corresponding author upon request.
